The article "The Effect of Fine-Grained Control of Workflow on Informal Learning: The Mediating Effect of Teacher Burnout" was retracted in 2024. Reasons: signs of a paper mill; suspected computer-generated content; unreliable results or conclusions; lack of ethics approval or compliance.

# The Effect of Fine-Grained Control of Workflow on Informal Learning: The Mediating Effect of Teacher Burnout

**DOI:** 10.1155/2022/3479295

**Published:** 2022-06-13

**Authors:** Zenghui Lu, Yanning Chen

**Affiliations:** Youjiang Medical University for Nationalities, Baise, Guangxi, China

## Abstract

Workflow fine control is an important research tool for the mediating effect of teacher burnout. Based on the fine control theory of workflow, this paper constructs a mediating effect model of teacher burnout in primary and secondary school teachers from the perspective of informal learning. The model designs a measurement scale based on the results of fine control, and the scale is revised through informal learning pretests to form the logical frame analysis loop of this paper. The scale uses Likert 5-point scoring, from 1.5 to represent never, rarely, occasionally, often, and always, which solves the difficulty of quantitative analysis of teacher burnout data. During the simulation process, SPSS 20.0 and AMOS 7.0 were used to conduct empirical analysis, exploratory factor analysis and confirmatory factor analysis on the survey data, and the measurement scales were tested. The empirical analysis results show that this paper uses cluster sampling and random sampling to carry out a questionnaire survey on 1022 primary and secondary school teachers. The measurement scale includes 19 items. Through exploratory factor analysis and confirmatory factor analysis, the control method is determined. In two dimensions, the revised control style questionnaire has a reliability of 0.951, and items with factor loadings less than 0.5 are eliminated, which effectively improves the control performance of informal learning.

## 1. Introduction

With the development of the information age, teachers will spend more and more time at work because of assistive technologies; as enterprises put forward higher and higher requirements for teachers, the phenomenon of job burnout is also gradually increasing [1–4]. Because the long-lasting negative effects of job burnout will far outweigh the positive effects, teachers' recovery time will also be deprived of job burnout. At present, most of the research in this field only stays in theoretical reasoning and assumptions, lacking the strong support of empirical research, and the cognition of perfectionists is often the premise of their behavior [5–7]. Therefore, this paper attempts to explore the relationship between perfectionism and job burnout from a cognitive perspective and investigate the relationship between different dimensions of perfectionism and job burnout in the context of regional culture, which will help enrich and improve the mechanism of job burnout formation.

Learning theory believes that intervention strategies should focus on the situational factors that reinforce the tendency of job burnout but ignores factors such as cognition, motivation, and emotion behind individual behavior; cognitive theory believes that intervention strategies should focus on the irrational values of job burnout but ignores the environmental factors that affect their cognitive concepts [8–11]. The causes of job burnout are multifactorial, and some scholars have begun to pay attention to the mechanism between various factors and job burnout. All in all, many phenomena show that the relationship between many factors and job burnout is not a simple connection.

The mediating effect test shows that transformational leadership can indirectly and directly have a positive predictive effect on teacher burnout, and the school organizational burnout atmosphere plays a partial mediating role. In terms of the duration of the mediation effect of teachers, the job burnout level of teachers with the mediation effect duration of less than 5 years, 6-10 years, and 11-15 years is significantly higher than that of teachers with the mediation effect duration of more than 21 years. There is a significant positive correlation, and the product-difference correlation coefficient is 0.563-0.588, which is higher than 0.298-0.382 for informal learning; the same school organizational burnout atmosphere and teacher burnout and its subdimensions also show a significant positive correlation; on the premise of excluding the influence of control variables, the regression analysis of informal learning found that the R2 value of transformational leadership in predicting teacher burnout was 0.386, and the *β* value of the standardized informal learning regression coefficient was 0.615. This study sheds light on the linking mechanisms between different dimensions of perfectionism and work addiction, attempts to explore how perfectionists avoid the negative effects of work addiction in a society where emerging technologies are constantly evolving, and refines the relationship between perfectionism and work addiction.

## 2. Related Work

Domestic scholars put forward that job burnout is the creation and job burnout of teachers in the teaching process. By applying the latest teaching and research results to teaching practice, teachers can generate unique insights and discover and apply new teaching methods [12–14]. Based on the elaboration of various scholars on job burnout, and referring to the definition, this paper believes that teacher burnout refers to the teaching goal of cultivating students' job burnout quality and job burnout ability in the process of teaching and actively and continuously adopting innovations created by others or themselves. Teaching philosophy, updating teaching content, adjusting new teaching methods and means in time, adopting new teaching resources and tools, improving teaching evaluation methods, and continuously improving teaching effect are a comprehensive teaching practice activity.

Bryant et al. [15] studied the relationship between perfectionism, job burnout, and job burnout among senior teachers of workflow and found that job burnout was positively correlated with perfectionists' personal standards and perfectionistic attention to mistakes. This questionnaire avoids the parental expectations and parental criticism dimensions of Cox's [16] perfectionism questionnaire, and after analyzing the positive aspects of perfectionism, it is changed to negative stereotypes about past perfectionism so that the questionnaire contains positive perfectionism and negative perfectionism. The two dimensions of perfectionism, at the same time, provide new diagnostic and evaluation tools for psychological counseling about perfectionism and provide new evidence for cross-cultural research on perfectionism. Furthermore, research by Carpenter and Green [17] showed that job burnout played a mediating role in the relationship between perfectionism (focus on mistakes) and burnout (fatigue), suggesting that job burnout plays a role in the relationship between perfectionism and burnout to a certain extent relationship.

Taking regional college students as a research sample, Tsai et al. [18] revised Frost's scale and finally obtained five dimensions: worry about mistakes, organization, parental expectations, personal standards, and doubts about actions, a total of 27 items; five dimensions in the Cronbach's alpha coefficients ranged from 0.64 to 0.81, and the test-retest reliability ranged from 0.63 to 0.82. The researchers revised the multidimensional perfectionism scale developed by Frost in the context of regional culture, and the results showed that parental criticism was not suitable for regional culture and divided FMPS into two factors, positive and negative, in which positive perfectionism included personal standards and organization, and negative perfectionism includes focusing on errors, parental expectations, and action anxiety [19–21]. The test-retest reliability of positive perfectionism and negative perfectionism is 0.81 and 0.79, respectively; the test-retest reliability of the total scale is 0.83, which indicates that the scale has good stability across time [22–25].

## 3. Workflow Granular Control Behavioral Metrics

### 3.1. Workflow Dependencies

Learning values are the independent variables of the workflow (denoted by *X*), learning adaptability is the dependent variable of the workflow (denoted by *Y*), and the mediating variable is the fine-control learning strategy (denoted by *M*). The informal learning regression coefficient of the dependent variable and the independent variable is denoted by *c*, the informal learning regression coefficient of the intermediate variable and the independent variable is denoted by *a*, the informal learning regression coefficient of the dependent variable and the mediating variable is denoted by *b*, and *c*′ is that when both independent and mediating variables are introduced into the regression equation, the independent and dependent variables are informally learned to change the regression coefficients.

(1) $$\begin{array}{c} \text{gertist}\left(m,n\right)=g\left(m\right)g\left(n\right)-\frac{g\left(m\right)}{1-g\left(m\right)}-\frac{g\left(n\right)}{1-g\left(n\right)}. \end{array}$$

Assuming that the correlation between *Y* and *X* is significant, it means that the informal learning regression coefficient *C* is significant. Under this premise, the intermediary variable *M* can be considered, and then, the coefficients *a* and *b* are tested in turn. If both are significant, it means that the influence of *X* on *Y* is at least part of this is achieved through the mediator variable *M*. At this point, look at the coefficient *C*′. If it is significant, it means that it is a partial mediating effect; that is, only a part of the influence of *X* on *Y* is realized by the mediating variable *M*. If it is not significant, it means that it is a complete mediating effect, and the influence of *X* on *Y* is completely achieved through the mediating variable *M*.

(2) $$\begin{array}{c} \left\{\begin{array}{c} \overset{i+k-1}{\underset{i=1}{\sum }}f\left(i,j\right)+f\left(k+i-j\right)=1,\\ \overset{i+k-2}{\underset{i=1}{\sum }}f\left(k\right)+f\left(k+i+j\right)=1. \end{array}\right. \end{array}$$

When establishing an informal learning regression model, if at least one of the coefficients *a* and *b* is not significant, the Sobel test needs to be done. Only when the Sobel test results are also significant can the mediating effect be significant. Using the Bootstrap method, 1000 samples were randomly selected with repeated repetitions, and the estimated value of 1000 coefficient products was obtained, 50% was used as the point estimate, and the 2.5%-97.5% estimated value constituted the 95% confidence interval of the point estimate. If the 95% confidence interval does not include “0,” it proves that the coefficient product is significant, and the mediating effect exists.

(3) $$\begin{array}{c} \overset{i+k-2}{\underset{i=1}{\sum }}1+f\left(k+i-j\right)\overset{i+k-1}{\underset{i=1}{\sum }}f\left(i,j\right)=1-f\left(k+i+j\right). \end{array}$$

For people with job burnout, on the one hand, job burnout has a direct positive effect on learning adaptability (*t* = 0.27, *P* < 0.001; 13 = 0.15, *P* < 0.001); that is, self-esteem person with high score of enterprising burnout has a higher level of learning adaptability. According to the viewpoint, testing a moderated mediation model requires estimates of the parameters of the three regression equations. All predictors were normalized in each equation. The research results show that perfectionism positively predicts work addiction, non-working-time assistive work technology positively predicts work addiction, and the interaction term between perfectionism and non-working-time assistive work technology has no significant predictive effect on work addiction.

(4) $$\begin{array}{c} \left\{\begin{array}{c} \text{rel}\left(x,y\right)=\max\left(x,y\right)-x,\\ \text{rel}\left(x\right)=\max\left(x\right)-\max\left(1-x\right). \end{array}\right. \end{array}$$

On the other hand, they have an indirect positive effect on learning adaptability through their own planning strategies and supervision and inspection strategies. That is, people with high self-esteem scores use less self-planning strategies and less supervision and inspection strategies and the higher the level of learning adaptability; people with high scores of enterprising burnout use less self-planning strategies, more supervision and inspection strategies, and better learning ability in higher adaptability.

### 3.2. Definition of Fine-Grained Control Methods

The fine control method mainly evaluates the suitability of measurement items. Commonly used item measurement methods include the homogeneity test method and the extreme group test method. The homogeneity test method is tested by the correlation coefficient of each item of the scale and the total score of the scale and the *α* coefficient of internal consistency of the scale; the extreme group test method is tested by the independent sample *T* test degree of the high and low groups of the scale, and the *T* value is used as the critical ratio or decision value (CR value) of the item; the larger the *T* value and the level of significance, the better the discrimination of the scale, and the decision value that does not reach the level of significance will be deleted. The results show that irrational beliefs in the workplace positively predict work addiction, and off-hour assistive work techniques positively predict work addiction. Prediction of addiction was significant. Therefore, Equation (5) satisfies the condition.

(5) $$\begin{array}{c} \text{armetuer}\left(p\left(x,y\right)\left|\left(x,y\right)\right.=\left(1,1\right)\right)=p\left(x\right)p\left(y\right)-\frac{1}{f\left(x,y\right)}. \end{array}$$

At the same time, observe that the correlation coefficient between the items and the total scale should preferably be above 0.30 and reach a statistically significant level; if the correlation coefficient between the corrected item and the total score is too small, or the coefficient suddenly increases after a certain item is deleted, it means that the case deleted this question.

(6) $$\begin{array}{c} j\left(\text{theta},t\right)=\text{aermu}\max\left(\log\overset{i+k-1}{\underset{i=1}{\sum }}q\left(t-\text{theta}\right)-\log\overset{i+k-1}{\underset{i=1}{\sum }}p\left(t+\text{theta}\right)\right). \end{array}$$

Informal learning can predict 14.1% of the variance of teachers' teaching burnout, and the standardized regression coefficients of contingent rewards, passive exception management, and active exception management are 0.375, 0.154, and 0.166, respectively, and reach a significant level; school organizational burnout atmosphere can predict that the burnout has 66.8% variation; transformational leadership can predict 66.2% variation of school organization job burnout climate, which is higher than the 35.3% variation of informal learning in Table 1. Correlation analysis was carried out on the variables involved in this study, and the mean, standard deviation, and correlation coefficient of each variable were displayed. It can be seen that the correlation between the variables has reached a significant level.

During the first exploratory factor analysis of the control scale, it was found that the items ICl, IC2, and IC3 had double loadings, and the factor loading values all exceeded 0.50, so they were deleted; the item IC3 factor loadings and the value are lower than 0.50; therefore, delete these two items. In the end, a total of two factors were extracted and named as “formal control” and “informal control,” which were quite different from the expectations when the questionnaire was designed in this paper. On the one hand, lightheartedness and family maintenance have a direct positive effect on learning adaptability (*B* = 0.33, *P* < 0.001; *B* = 0.19, *P* < 0.001); that is, lightheartedness and family maintenance score high, the higher the learning adaptability.

(7) $$\begin{array}{c} \text{wertist}\left(\text{in},\text{out}\right)=\frac{1-\text{in}\left(x\right)}{1-\text{out}\left(t\right)}-\text{padding}\left(x\left[1:i\right]-x\left[-i:1\right]\right)-1. \end{array}$$

It can be seen that in the two-dimensional model, each index is within the standard range, where *χ*2/df is 1.517 less than 2; RMR is 0.043 and less than 0.08; RMSEA = 0.044 < 0.05; GFI, AGFI, CFI, and IFI are all greater than 0.90; these indicators indicate that the two-dimensional model has a good goodness of fit. Therefore, the 2D model of the control mode is very well validated.

### 3.3. Informal Learning Factor Iteration

Principal component analysis and Varimax orthogonal rotation method were used for the 13 items of the school teachers' burnout behavior scale to explore the informal learning factor dimension of school teachers' burnout behavior, and finally, two factors were extracted, the first one. The factor is named “job burnout idea generation,” and the second factor is named “job burnout idea execution,” which is also consistent with the research results of scholars such as it. The analysis results of the mediation effect are as shown, with positive perfectionism as the independent variable and coworker approval and work addiction as the dependent variables, respectively; the results show that the confidence interval does not contain “0,” and the mediation effect is significant.

(8) $$\begin{array}{c} \text{kenel}\left(x,y\right)-\text{size}\left(x,y\right)=\frac{\text{size}‐\text{wertist}\left(\text{in},\text{out}\right)}{1‐\text{wertist}\left(\text{in},\text{out}\right)}-\text{wertist}\left(1‐\text{kenel},1+\text{kenel}\right). \end{array}$$

As shown in below, the factor loading of each item is greater than 0.50, and the two obtained factors cumulatively explain 75.094% of the variation, and there is no cross-loading between each item, indicating that the questionnaire is effective. The degree of accuracy is good, and the meaning of each variable can be accurately measured.

Figure 1 uses the Amos 7.0 software for confirmatory factor analysis, and the analysis results are shown. It can be seen from it that in the two-dimensional model, all indicators are within the standard range, in which the chi-square degree of freedom (*χ*2/df) is 1.646 less than 2, and the residual root mean square is 0.055 and less than 0.08, and the root mean square error of approximation (SEA) = 0.056, which is between 0.05 and 0.1, indicating that the model is in the gray area, which is acceptable, and the goodness of fit index (GFI), adjusted goodness-of-fit index (AGFI), comparative fit index (CFI), and incremental fit index (QI) were all greater than 0.90. This standard and these indicators all indicate that the two-factor model has a good goodness of fit. Therefore, a two-dimensional model of school teachers' burnout behavior is supported by the data.

(9) $$\begin{array}{c} \left\{\begin{array}{c} \overset{i+k-1}{\underset{i=1}{\sum }}w\left(i,j\right)\cup w\left(i,i-h-1\right)=1,\\ \overset{i+k-1}{\underset{i=1}{\sum }}y\left(i,j\right)\cup y\left(i,i-h-1\right)=1. \end{array}\right. \end{array}$$

It can be seen that the difference of age on the level of not holding an administrative position is extremely significant (*F* = 3.964, *P* = 0.009), which indicates that the negative emotion scores of different age groups on the level of not holding an administrative position are different and extremely significant; but the difference was not significant in the level of holding administrative positions (*F* = 1.028, *P* = 0.387). After a simple and simple effect analysis, the negative emotion scores of teachers who do not hold administrative positions over the age of 150 are significantly higher than those of 430-year-old teachers (0.032) and 3-40 years old (0.002), 4 to 50 years old (0.045); teachers aged ≤ 30 years old were significantly higher than those of 31-40 years old (0.013).

## 4. Construction of the Mediation Effect Model of Teacher Burnout Based on Fine Control of Work Process

### 4.1. Workflow Dimension Distribution

According to the analysis method of the mediation effect of the informal learning factor, the Bootstrap method is used, and 5000 samples are randomly selected with replacement, and the estimated value of 5000 coefficient products is obtained, and 50% is used as the estimated value of the workflow dimension point; 2.5%-97.5% estimate constitutes the 95% confidence interval for the point estimate. If the 95% confidence interval does not include “0,” it proves that the coefficient product is significant, and the mediating effect exists.

(10) $$\begin{array}{c} \left\{\begin{array}{c} p\left(x,y\right)=\frac{1-p\left(x\right)/p\left(y\right)}{1+p\left(x\right)/p\left(y\right)},\\ r\left(x,y\right)=\frac{1-fp\left(x\right)/fp\left(y\right)}{1+fp\left(x\right)/fp\left(y\right)}. \end{array}\right. \end{array}$$

This paper uses the Bootstrap method to test the mediating effect of fine control in the workplace. Confirmatory factor analysis was performed on the four variables involved in the study using Amos 7.0, and an overall structural equation model was constructed to determine the fit of the overall model. The model fit index was as follows: *χ*2 was 156.530, *χ*2/df was 9.208, and RMSEA was 0.124; the model was acceptable.

(11) $$\begin{array}{c} \left[\begin{array}{c} \text{dialation}\left(t,t-1\right)*\text{kenel}\left(1-t,1\right)\\ \text{strike}\left[0,1,t-1,t\right] \end{array}\right]\in \left[\begin{array}{c} 1-\frac{fp\left(x\right)}{fp\left(y\right)}\\ 1+\frac{fp\left(x\right)}{fp\left(y\right)} \end{array}\right]. \end{array}$$

After a simple and simple effect analysis, it can be seen that the monthly salary income of teachers with overseas experience ≤ 3000 yuan is significantly smaller than the monthly salary income of 3001-4000 yuan (0.027), 4001-5000 yuan, and ≥5000 yuan (0.030) positive emotion score, because the higher the salary is, the more useful the knowledge is, so the positive emotion score is high. On the other hand, lightheartedness has an indirect positive effect on learning adaptability through self-planning strategies; that is, people with high scores of lightheartedness and happiness use more self-planning strategies, while the use of self-planning strategies affects learning adaptability and makes them adaptable to learning, the higher the level of sexuality.

(12) $$\begin{array}{c} \left[\begin{array}{cc} \frac{n-s\left(x,y\right)/2p\left(x,y\right)}{n-1} & p\left(x,y\right)-1\\ p\left(x,y\right) & \frac{p\left(x,y\right)}{s\left(x,y\right)} \end{array}\right]⟶\left[\begin{array}{cc} 1 & -\cos p\left(x,y\right)\\ \sin p\left(x,y\right) & -1 \end{array}\right]. \end{array}$$

Workflow construct validity refers to the degree to which a measurement tool can measure a concept or trait of a theory. This paper first uses the SPSS 16.0 software to conduct exploratory factor analysis (EFA) to explore the constituent dimensions of research variables and then uses the Amos 7.0 software to conduct confirmatory factor analysis (CFA) to analyze the factor model. The steps of exploratory factor analysis are as follows: first, it is necessary to explain the structure of the sample, the overall arrangement of the measurement, and the relationship between related aspects.

(13) $$\begin{array}{c} \left[\begin{array}{c} \text{padding}\left(x,1\right)\\ \text{padding}\left(-x,-1\right)\\ \text{padding}\left(x,-1\right)\\ \text{padding}\left(-x,1\right) \end{array}\right]\cup X\left(x\right)=R. \end{array}$$

This paper uses the KMO sample measure (Kaiser Meyer-Olkin Measure of Sampling Adequacy) to test the degree of correlation between the items which is combined with Bartlett's test of sphericity to judge whether it is suitable for factor analysis. If the KMO value and Bartlett's sphericity test results indicate that factor analysis is suitable, then the basic factors are isolated from several data to analyze the concept validity of the measurement. In this paper, KMO test and Bartlett sphericity test are firstly performed on the three variables of salesperson burnout behavior, control style, and self-efficacy to judge whether these three variables are suitable for factor analysis. For the specific test results, it may see the text.

### 4.2. Fine Control Energy Efficiency Perception

Taking negative perfectionism as the independent variable of fine control energy efficiency, performance requirements, and job burnout as dependent variables, respectively, the research results show that the confidence interval does not contain “0,” and the mediating effect is significant. Testing the moderated mediation model requires estimating the parameters of the three informally learned regression equations. All predictors were standardized in each equation (Dearing and Hamilton). The results of the study are shown in Figure 2. For self-respecting, enterprising, and innovative people, on the one hand, self-respect and enterprising innovation have a direct positive effect on learning adaptability (0 = 0.27, *P* < 0.001; 13 = 0.15, *P* < 0.001); that is, people with high scores of self-respect and enterprising innovation have a higher level of learning adaptability.

Secondly, the main effect of fine control energy efficiency was analyzed (*F* = 9.16, *P* < 0.001). After the postmortem test, it was found that the first grade (MD = 6.68, HS = 0.001; MD = 3.13, 0.01; MD = 6.28, *P* < 0.001; MD = 8.70, *P* < 0.001) the level of relaxed and happy learning of students was significantly higher than that of junior three, senior one, senior two, and senior three: the level of relaxed and happy learning of the students in the first grade (MD = 3.56, *P* < 0.001; MD = 3.15, *P* < 0.01; MD = 5.57, *P* < 0.001) was significantly higher than that of the first graders 3. For the students of senior two and senior three, the level of relaxed and happy learning of senior two (MD = 2.42, *P* < 0.05) was significantly higher than that of senior three.

On the other hand, they have an indirect positive effect on learning adaptability through their own planning strategies and supervision and inspection strategies. That is, people with high self-respect scores use less self-planning strategies and less supervision and inspection strategies and the higher the level of learning adaptability; people with high scores of enterprising innovation use less self-planning strategies and more supervision and inspection strategies and learn to adapt. There was no significant difference between the third year of junior high school and the second and third years of senior high school. From a statistical point of view, the mood of relaxed and happy learning in the third and senior years is significantly lower than that of the first, senior, and senior two; that is, compared with the graduating class, students in other grades have more relaxed and happy learning levels.

After the factor analysis of Figure 3, its reliability and validity should be tested, that is, the reliability test of the scale. Reliability can also be regarded as the degree to which the measurement results are affected by measurement errors. In this paper, the Cronbach and coefficient are used to test the internal consistency reliability coefficient of the scale. When the Cronbach and coefficient are higher, the reliability of the scale is higher. According to standard division, the Cronbach and coefficient of the factor level are better when it is greater than 0.7, and it is barely acceptable between 0.6 and 0.7; the coefficient of the total scale is better than 0.8, and the reliability is better when it is greater than 0.9. Fine control in the workplace positively predicts job burnout, nonworking time assistive work technology positively predicts job burnout, and the interaction term between fine control and nonworking time assistive work technology in the workplace is a significant predictor of job burnout. Therefore, it satisfies the condition.

### 4.3. Evaluation of the Mediating Effect of Job Burnout

The scale uses the improved mediation burnout scale (DUWAS), which includes two subscales: forced work (for example, "I often feel that something in my heart forces me to work hard") and overwork (for example, "I feel that work is like a race against time").The two subscales each have 5 items, which are scored on a 5-point Likert scale, ranging from 1 to 5, representing “completely inconsistent” to “completely consistent.” This paper conducts a confirmatory factor analysis on the scale, and the results are shown in Figure 4. The scale's Cronbach's alpha coefficient was 0.877. Taking negative perfectionism as an independent variable and colleagues' recognition and job burnout as dependent variables, the results show that the confidence interval does not contain “0,” and the mediating effect is significant. A revised Work Communication Tool Use Scale was used, consisting of 3 items. The scale's Cronbach's alpha coefficient was 0.822.

The study in Figure 4 selected demographic data such as region, gender, and grade to examine the developmental characteristics of middle school students' fine-control learning strategies. First, taking the scores of the four fine-control learning strategies as the dependent variable and taking the region, gender, and grade as the independent variables, the fine-control learning strategies of middle school students were evaluated by 2 (rural students, urban students) × 2 (male, female) × 5 (primary school students). The multivariate analysis of variance of the third year of junior high school, the first year of senior high school, the second year of senior high school, and the third year of senior high school is used to analyze the development characteristics of the fine control learning strategy of middle school students. First, the main effect of grade was analyzed (*t* = 5.77, *P* < 0.001). 12 factors were explored, some of which had 2 or one topic, and could not be combined with other factors, so such topics were deleted, and the small factor load items were deleted. According to the scree plot, 9 factors were finally retained. It is more appropriate, the questionnaire is omitted, a total of 16 questions are eliminated, and 53 questions are reserved. The results of factor analysis are as follows:

(14) $$\begin{array}{c} \left\{\begin{array}{c} y\left(i\right)-ax\left(i\right)-b=\sin\left(i\right)-ax\left(i\right)-\cos b=0,\\ y\left(j\right)-ax\left(j\right)+b=\cos\left(j\right)-ax\left(j\right)+\sin b=1. \end{array}\right. \end{array}$$

The post hoc test of grades found that the first year of junior high school (MD = 7.29, *P* < 0.001; MD = 4.28, *P* < 0.01; MD = 5.86, *P* < 0.01; MD = 10.32, *P* < 0.001) grade family maintenance was significantly higher than that of junior three, senior one, senior two, and senior three; senior one (*t* = 6.30, *P* < 0.01; MD = 8.21, *P* < 0.001) grade family maintenance is significantly higher than that of the third year of junior high school and the third year of senior high school. There is no significant difference between the first grade and senior grade 1: there is no significant difference between the third grade and senior grade 3; that is, the lower grade students of the junior high school and senior high school are more inclined to think that learning is for the values of family maintenance than the students in the senior grade of the junior high school and senior high school.

(15) $$\begin{array}{c} \frac{\sqrt{\mathrm{var}\text{riation}\left(x,t\right)-1}}{\mathrm{var}\text{riation}\left(x,t\right)}+\frac{\sqrt{\mathrm{var}\text{riation}\left(y,t\right)-1}}{\mathrm{var}\text{riation}\left(y,t\right)}+\frac{\sqrt{\mathrm{var}\text{riation}\left(z,t\right)-1}}{\mathrm{var}\text{riation}\left(z,t\right)}=1. \end{array}$$

Content validity, also known as face validity and logistic validity, refers to whether the measurement tool used can cover all the items (levels) of the content it is intended to measure. The scales used in this paper are, on the one hand, translated from foreign mature measurement scales, and, on the other hand, revised and improved through interviews and preinvestigations to form the final measurement scale. Therefore, the overall scale of this paper has good content validity.

Take men and women as two dimensions of interdependence, that is, men's use of work communication tools and women's use of work communication tools as two dimensions of interdependence. Through confirmatory factor analysis, it was found that the results were as follows: *χ*2 = 9.85, df = 5, RMSEA = 0.042, and TLI and CFI and other indicators were up to the standard. It can be seen from the above that the construct validity and reliability of the scale meet the requirements of psychometrics. The factor analysis of the scale shows that the KMO sampling appropriateness measure is 0.964, and the *X* value of the Bartlett sphericity test is 5036.409, which reaches a significant level, indicating that there is a common factor between the overall correlation matrices, which is very suitable for factor analysis.

### 4.4. Analysis of Informal Learning Variables

The informal learning scale includes two dimensions: positive perfectionism and negative perfectionism, 25 items (12 items for positive perfectionism, 13 items for negative perfectionism), using Likert 5-point scoring, 1-5 corresponding to no, somewhat, appropriately, quite a lot, and very much. The higher the score, the more positive or negative perfectionism tendencies are as shown. The scale's Cronbach's alpha coefficient was 0.933. Validity refers to the question of correctness, which refers to whether the results measured by the measurement tools used can reflect the true degree of what the researchers want to measure. The results of confirmatory factor analysis on the questionnaire data using the LISREL 8.70 software can also illustrate the construct validity of the questionnaire.

The principal component analysis method and orthogonal rotation with the Varimax method in Figure 5 are used to obtain the loading value of each informal learning factor, and the items with the loading greater than 0.5 are retained, and the eigenvalue is greater than or equal to 1 as standard factor extraction. After convergence after several iterations, 4 items of the double-load phenomenon were deleted, and the cumulative variance contribution rate was 80.944%. A total of four factors were distinguished, and the results were roughly in line with expectations. Observing the item analysis results of informal learning, it can be found that the decision values of all items have reached a significant level, and the correlation coefficient between the items in the homogeneity test and the total scale is between 0.423 and 0.578, after the items are deleted. Except for JY11, there is no sudden increase in the *s* coefficient, so it is necessary to delete the item JY11. It can be seen that the mediating effect of supervision and inspection strategies on the relationship between self-confidence and independence and learning adaptability is relatively large, while the mediating role of self-planning strategies in the relationship between self-esteem and learning adaptability is relatively small.

(16) $$\begin{array}{c} \left\{\begin{array}{c} \forall \overset{i+k-1}{\underset{i=1}{\sum }}x\left(i\right)\left|\bar{x\left(i\right)-x\left(0\right)}\right|+y\left(i\right)\left|\bar{u\left(i\right)-u\left(0\right)}\right|>1,\\ \exists y\left(i\right)+x\left(i\right)>1. \end{array}\right. \end{array}$$

In order to test the influence of control method on the job burnout behavior of school teachers, a linear relationship was found between the control method and the job burnout behavior of school teachers through the scatter plot. Therefore, the regression analysis of informal learning is carried out with the two-dimensionality of the job burnout behavior of school teachers as the dependent variable and the formal control and the informal control as the independent variables.

(17) $$\begin{array}{c} \left[\begin{array}{c} \overset{i+k-1}{\underset{i=1}{\sum }}\log\left(i-1\right)\\ 1-\overset{i+k-1}{\underset{i=1}{\sum }}q\left(i-1\right) \end{array}\right]+\left[\begin{array}{c} \overset{i+k-1}{\underset{i=1}{\sum }}\log\left(i+1\right)\\ 1-\overset{i+k-1}{\underset{i=1}{\sum }}q\left(i+1\right) \end{array}\right]<\left[\begin{array}{c} \overset{i+k-1}{\underset{i=1}{\sum }}\exp\left(i-1\right)\\ 1-\exp\left(i\right) \end{array}\right]. \end{array}$$

The informal learning regression analysis results are shown in it. Among them, the variance inflation factor VW of the independent variable is 1.079, which is far less than 10, and the tolerance is 0.927, which is much higher than the conventional limit of 0.10, which indicates that the white variable does not have serious collinearity problem, which meets the assumptions of linear informal learning regression.

## 5. Application and Analysis of the Mediation Effect Model of Teacher Burnout Based on Fine Control of Workflow

### 5.1. Workflow Data Output

Naming the first workflow data dimension as “colleague approval” to explain those items that require approval and support from colleagues, including items 14, 15, 16, 17, and 18, and name the second dimension as “Failure” is used to explain the items of fear of failure and avoidance of failure, including items 19, 20, 21, 22, 23, and 24, and the third dimension is named “performance requirements” to explain the pursuit of better high performance; set the items of performance requirements for yourself, including items 9, 10, 11, 12, and 13, and named the fourth dimension “control” to explain employees' sense of job control at work. The items included are 25, 27, and 28. In confirmatory factor analysis, the scale of Figure 6 had a Cronbach's alpha of 0.901.

The results of analyzing the 77 items of the prediction questionnaire show that the CR values of items 1, 5, 6, 7, 17, 18, 24, 32, 34, 65, and 85 in this questionnaire did not reach their significant level. This item should be deleted, and the CR values of the remaining items are extremely significant (*P* < 0.05), indicating that they have good discriminating power and are suitable for retention. Next, further exploratory factor analysis will be conducted on the 66 items. The KMO value of the informal learning scale is 0.870. The closer the KMO value is to 1, the more common factors between variables, the more suitable for factor analysis. It is the rotated factor matrix, which is orthogonally rotated by the Varimax rotation method, and the Kaiser normalization method is used during rotation, and it undergoes multiple iterative conversions during rotation. The cumulative contribution rate of the factors is 70.194%.

Under the conditions of controlling the influence of factors such as region, gender, and grade, this paper studies seven learning values: lightheartedness, self-respect, social development, self-development, enterprising innovation, family maintenance, and self-confidence and independence. There are significant differences in the impact of learning adaptability (*a* = 0.34, *P* < 0.001; *a* = 0.27, *P* < 0.001; *a* = 0.28, *P* < 0.001; *a* = 0.12, *P* < 0.001; *P* < 0.001; that is, the regression coefficient *c* is significant): while the self-planning strategy and the supervision and inspection strategy have a significant impact on learning. Adaptability has a significant effect (*L* = 0.02, *P* < 0.01: *L* = 0.02, *P* < 0.001; that is, the regression coefficient *b* is significant). The results show that the eigenvalues of the three common factors in Figure 7 are all between 0.50 and 0.90, and the cross-loading situation is excluded, which has good convergent and discriminant validity.

The differences in the workflow between genders at the age of 30-40 were extremely significant (*F* = 12.115, *P* = 0.001), which indicated that the differences in the positive emotion scores of different genders at the age of 3-40 were extremely significant. From the mean point of view, the score of male students (*M* = 3.511) was significantly higher than that of female students (*M* = 2.903). Male teachers between the ages of 31 and 40 are in a period of rising careers, and their basic families will be very stable, while women are faced with various things such as marriage, childbirth, and work.

It is generally believed that the smaller the model, the better the fit, and the index is greatly affected by the sample size, so it is of little significance: for CFI and NNFI, the larger the value, the better; it is generally believed that it should be greater than 0.90, and some people think that it should be greater than 0.80; the model is basically acceptable. For RMSEA, Steiger believes that RMSEA is lower than 0.1 means a good fit, below 0.05 means a very good fit, and below 0.01 means a very good fit.

### 5.2. Fine-Controlled Informal Learning Simulation

First, the item analysis of the fine control data shows that the total correlation coefficient is 0.322, which is less than 0.4, so the 26th question is deleted. On this basis, exploratory factor analysis was performed on the remaining items, and the results showed that the KMO value was 0.884, and the Bartlett sphericity test value was 1707.239 (df = 190, *P* = 0.000), indicating that the scale is suitable for factor analysis. Using the principal component analysis method and the Kaiser standardized optimal skew method, the scale finally formed 4 dimensions, a total of 19 items, and the cumulative interpretation rate was 70.323%, and the 27 dimensions of the research process were named. The results of an exploratory factor analysis of fine control in the workplace are shown. There was only a significant main effect of gender type in self-esteem (*F*(1,492) = 3.67, *P* < 0.05). After the postmortem analysis, it was found that the level of self-esteem of girls (*H* 3.26, SD = 0.70) was significantly higher than that of boys (*M* = 3.06, SD = 0.78), indicating that compared with boys, girls are more inclined to learning is for self-respect.

From the factor analysis results of the teacher burnout scale, it is found that five main factors can be extracted from the 25 test items through the main axis extraction method. They are 19.093%, 17.869%, 15.561%, 14.786%, and 8.971%, respectively, and the eigenvalues are all greater than 1. The basic assumptions of each test supporting factor analysis are not violated, and all items also have a considerable degree of appropriate sampling, indicating that the scale items have considerable homogeneity; the Cronbach's coefficient of the total scale is 0.975, reflecting that the reliability of the scale in Figure 8 is good.

The results of the confirmatory structural model analysis of the school organization job burnout climate scale are shown in the following table, because some of the fitting indicators obtained from the first test did not meet the adaptation standard, and the revised index value was greater than 5, indicating that the releases meet the fitting criteria, and other value-added fit indices are all above 0.90, indicating that the model fitting situation after release is lower than that before parameter release. The chi-squared degrees of freedom ratio is between 1 and 5, the asymptotic residual mean square sum square root RMSEA is less than 0.08, the fitness index GFI is greater than 0.90, the residual mean square sum square root RMR is less than 0.05, and the incremental fitness indexes TLI, CFI, and IFI are greater than 0.90, indicating that the structural model of the teacher burnout scale fits the data better. In this study, the reliability of each subscale of the questionnaire was 0.81 for physical and mental health and 0.81 for learning ability, the learning environment is 0.80, the friendship relationship is 0.84, and the *a* coefficient of the total questionnaire is 0.89. The results of verification factor analysis are as follows: threat 3.06, NNFI = 0.92, CFI = 0.90, and RMSEA = 0.06, indicating that the data supports the model construct.

Taking formal control and informal control as fine control independent variables and self-efficacy breadth as the dependent variable in Figure 9, a multivariate informal learning regression analysis was conducted. The *F* value of the model is 7.292, and the significance level is 0.009, indicating that the model fits well. The results of the regression analysis of informal learning showed that both formal control and informal control had a significant positive effect on the breadth of self-efficacy (*s* = 0.102, *P* < 0.05; *t* = 0.048, *P* < 0.1); hypothetical H7c and hypothetical H8c are supported. In this model, the adjusted R2 is 0.060, indicating that the control method explains 6.0% of the change in the self-efficacy breadth. It can be considered that the control method has a certain degree of influence on the teacher's self-efficacy breadth.

### 5.3. Example Application and Analysis

Fine-control scores were measured using a 5-point Likert scale, with higher scores indicating more frequent use of assistive work technology during nonworking hours. The scale's Cronbach's alpha coefficient was 0.822. Confirmatory factor analysis found that the results were as follows: *χ* = 9.85, df = 5, RMSEA = 0.042, and TLI and CFI and other indicators were up to standard. It can be seen from the above that the construct validity and reliability of the scale meet the requirements of psychometrics. Judging from the reliability of the results, the reliability of the seven dimensions has reached more than 0.70, and the overall reliability is 0.93, indicating that the questionnaire has good reliability and can be used for future research in related fields.

From the distribution of the mediation effect period, it can be seen that teachers with a mediation effect period of less than 5 years and more than 21 years account for 25.7% and 20.7%, respectively, followed by teachers with a mediation effect period of 6-10 years also occupy a larger proportion in Figure 10; the duration of the intermediary effect of the surveyed primary and secondary school teachers shows a trend of bipolar distribution; in terms of teacher education distribution, undergraduate education has become the main component of the surveyed teachers, followed by the proportion of teachers with college education and below is 25.1%, and the proportion of teachers in the sample schools is relatively reasonable.

The formats of text and data charts are distinguished: the meanings of text and data charts correspond to the following, and one of the dimensions is used as the evaluation of self-regulation learning strategies, and confirmatory factor analysis of the scale is carried out. The fitting index is good, indicating that the self-regulated learning strategy questionnaire has good construct validity. The self-efficacy intensity of the mediating variable in Table 2 has a significant impact on the dependent variable school teacher job burnout concept (*t* = 0.309, *P* < 0.01), and the independent variable formal control and informal control have a significant impact on the dependent variable salesperson job burnout. The effect of behavior was significant (S3.1 = 0.118, *P* < 0.05; B3.2 = 0.165, *P* < 0.01). The process of analyzing the mediating effect of self-efficacy is shown in it below. It can be seen from the table that the S3.1 value of the formal control of the independent variable in the third step is smaller than the B1.1 value of the independent variable in the first step (0.118 < 0.136), so the strength of self-efficacy is in the formal control. There is a mediating effect between control and the conception of job burnout of school teachers; the S3.2 value of informal control in the third step is smaller than the S3.3 value of the independent variable in the first step (0.165 < 0.219); therefore, the strength of self-efficacy has a partial mediating effect between informal control and the conception of school teachers' job burnout.

## 6. Conclusion

This paper constructs a mediating effect analysis model based on the elements of formal control and job burnout. Self-efficacy strength and self-efficacy breadth both have partial mediating effects between informal control and the implementation of school teachers' job burnout concept. Hypothesis H12 is also partially supported. Therefore, self-efficacy breadth has a partial mediating effect between formal control and the conception of school teachers' job burnout; the value of informal control in the third step is smaller than the value of the independent variable in the first step (0.205 < 0.219); therefore, self-efficacy breadth has a partial mediating effect between informal control and the conception of school teachers' job burnout. In this paper, the reliability of each subscale of the questionnaire is as followed: light-hearted is 0.91, self-esteem is 0.89, social development is 0.91, self-development is 0.72, enterprising innovation is 0.77, family maintenance is 0.78, self-confidence independence is 0.77, the total reliability of the questionnaire is 0.93, and the result of verification factor analysis is *zd*/df = 3.32, NNFI = 0.91, CFI = 0.91, and RMSEA = 0.05, indicating that the data supports the model construct. From the results of reliability analysis, the reliability of the four dimensions of the scale has reached 0.76 or more, and the reliability of the total scale has reached 0.7692, indicating that the fine control strategy scale has certain reliability and can be used in future research in related fields. There are still some shortcomings in this study. For example, this study used a cross-sectional design, which did not take into account the role of time factors that may affect its mechanism. In view of this, follow-up studies can deepen the study design and refine the influence mechanism of perfectionism on work addiction to make the study more ecologically valid.

## Figures and Tables

**Figure 1:** Informal learning factor iteration.

**Figure 2:** Confidence interval of fine control energy efficiency.

**Figure 3:** Analysis of fine control energy efficiency reliability.

**Figure 4:** Analysis of the mediation effect of job burnout.

**Figure 5:** Analysis of informal learning variables.

**Figure 6:** Workflow fine control coefficient distribution.

**Figure 7:** Workflow data output difference analysis.

**Figure 8:** Factor analysis of teacher burnout scale.

**Figure 9:** Fine control of informal learning dimension.

**Figure 10:** Construct validity and reliability of fine control subsection.

**Table 1:** Fine control prediction.

Fine control case	Stage 1	Stage 2	Stage 3
Variation *a*	39.65	71.90	12.70
Variation *b*	44.90	43.33	18.75
Variation *c*	77.04	76.38	82.36
Variation *d*	43.14	42.62	48.96
Variation *e*	11.34	88.06	18.59
Variation *f*	12.06	99.31	32.19
Variation *g*	38.75	55.34	34.57

**Table 2:** Teacher burnout mediating variable self-efficacy intensity.

Burnout case	Self-efficacy intensity	Concept 1	Concept 2	Concept 3	Concept 4
1	Variable salesperson	0.449	0.433	0.187	0.743
2	Burnout concept	0.770	0.764	0.824	0.022
3	Informal control	0.431	0.426	0.490	0.594
4	Formal control	0.113	0.881	0.186	0.375
5	Independent variable	0.121	0.993	0.322	0.382
6	Control and the conception	0.004	0.553	0.346	0.128

## Data Availability

The data used to support the findings of this study are included within the article.
